The article "Effect of Xinyi Biyan Pill in Adjuvant Treatment of Patients with Chronic Rhinosinusitis and Its Influence on Serum Inflammatory Factors and Immune Function" was retracted in 2023. Reasons: signs of a paper mill; compromised peer review; unreliable results or conclusions.

# Effect of Xinyi Biyan Pill in Adjuvant Treatment of Patients with Chronic Rhinosinusitis and Its Influence on Serum Inflammatory Factors and Immune Function

**DOI:** 10.1155/2021/2228803

**Published:** 2021-08-27

**Authors:** Qingfu Bao, Yu Zhou, Lei Zhang

**Affiliations:** ^1^Department of ENT & HN Surgery, Shao Yifu Hospital Affiliated to Medical College of Zhejiang University, Hangzhou, Zhejiang 310000, China; ^2^Department of ENT & HN Surgery, Zhejiang Hospital of Integrated Traditional Chinese and Western Medicine, Hangzhou, Zhejiang 310000, China; ^3^Department of ENT & HN Surgery, The 903th Hospital of PLA Joint Logistics Support Force, Hangzhou, Zhejiang 31000, China

## Abstract

**Objective:**

To explore the effect of Xinyi Biyan Pill in adjuvant treatment of patients with chronic rhinosinusitis (CRS) and its influence on serum inflammatory factors and immune function.

**Methods:**

From January 2017 to April 2020, 112 CRS patients admitted to this hospital were randomly divided into the control group (*n* = 52) and the study group (*n* = 60). The control group was treated with endoscopic sinus surgery (ESS), after the operation, levofloxacin capsules were taken orally, budesonide nasal spray was given, and the nasal cavity was flushed with normal saline; on the basis of that mentioned above, the study group was treated with Xinyi Biyan Pill orally after the surgery. The clinical efficacy and the symptom relief time of nasal congestion and runny nose, hyposmia, mucosal edema, and vesicles disappearance of the two groups after treatment were observed; the serum inflammatory factors' (C-reactive protein (CRP), interleukin-6 (IL-6), and interleukin-8 (IL-8)) and immune function indexes' (total immunoglobulin E (TIgE), eosinophil cationic protein (ECP), CD3^+^, CD4^+^, and CD4^+^/CD8^+^) expression levels before and after treatment in the two groups were detected; the recurrence of CRS after 1 year of treatment in the two groups was recorded.

**Result:**

After treatment, the total clinical effective rate of the study group (92.98%) was significantly higher than that of the control group (78.00%) (*P* < 0.05). After treatment, the symptom relief time of nasal congestion and runny nose, hyposmia, mucosal edema, and vesicle disappearance in the study group was shorter than that in the control group (*P* < 0.05). After treatment, the expression levels of serum CRP, IL-6, and IL-8 in the two groups were significantly lower than those before treatment, and the study group was significantly lower than the control group (*P* < 0.05). After treatment, the expression levels of serum TIgE and ECP of the two groups were significantly lower than those before treatment, the expression levels of serum CD3^+^, CD4^+^, and CD4^+^/CD8^+^ of the two groups were significantly higher than those before treatment, and the study group had significant changes compared with the control group (*P* < 0.05). After 1 year of treatment, the recurrence rate of CRS in the study group (1.79%) was significantly lower than that in the control group (12.00%) (*P* < 0.05).

**Conclusion:**

Xinyi Biyan Pill has a significant clinical effect in adjuvant treatment of CRS patients. It can effectively reduce the expression level of serum inflammatory factors, improve the body's immune function, and prevent short-term recurrence. It is worthy of clinical promotion.

## 1. Introduction

Chronic rhinosinusitis (CRS) is a chronic and complicated purulent inflammation commonly found in otolaryngology, with the nasal cavity and sinus mucosa as the main sites of disease. Its incidence in European and American adults is about 10% or more [1]. Patients often have local symptoms such as nasal congestion and runny nose, decreased sense of smell, facial pain, and head pain as clinical manifestations [2]. The disease usually develops from improper treatment or incomplete treatment of acute sinusitis, and if the treatment of CRS is not timely and standardized, the patient's condition will be prolonged, unhealed, and recurrent attacks for a long time, and it is also easy to induce other clinical complications such as nasal polyps and cranioocular pulmonary infection, which seriously affect the quality of life and life safety of patients [3, 4]. The pathogenesis of the disease is complicated, and its proinflammatory potential is enhanced, immune function declines, and tissue remodeling is closely related to its occurrence and development [5, 6]. For the treatment of CRS, in terms of surgical intervention, the removal of the patient's lesion site and the expansion of the nasal sinus opening with endoscopic sinus surgery (ESS) are important treatment methods, which are minimally invasive and have the effect of preserving the structure of the nasal cavity and its physiological functions to the greatest extent; however, it cannot completely control inflammation and enhance immune function when used alone, and it is still easy to relapse after surgery [7]; therefore, it must be combined with auxiliary methods such as drug treatment; at present, there are clinical treatments such as antibiotics, glucocorticoids, and immunomodulators; for example, the common macrolide antibiotics such as azithromycin can inhibit the production of inflammatory cytokines and the recruitment of neutrophils and improve the immune function and mucus quality; however, the side effects of such drugs and the interaction between drugs affect their long-term application [8, 9]. In recent years, Chinese medicine has made great progress in the research of chronic rhinitis, and its drug treatment effect has become more prominent. Xinyi Biyan Pill is an over-the-counter medicine for the clinical treatment of acute and chronic rhinitis or allergic rhinitis, which belongs to exogenous wind-heat syndrome, and it has the effects of dispelling wind and relieving internal heat or fever, detoxification inflammation, and detoxification. In recent years, our department has used Xinyi Biyan Pill for the adjuvant treatment of CRS patients after ESS and achieved satisfactory results. The specific report is given below.

## 2. Materials and Methods

### 2.1. General Information

From January 2017 to April 2020, 112 CRS patients admitted to this hospital were randomly divided into the control group (*n* = 52) and the study group (*n* = 60). This study was approved by the ethics committee. There was no statistical difference between the two groups of general information in Table 1 (*P* > 0.05) (comparable).

### 2.2. Inclusion Criteria

① Patients who met the diagnostic criteria of CRS in the “Canadian guidelines for chronic rhinosinusitis: Clinical summary” [10]. ② Patients who met the traditional Chinese medicine diagnostic criteria for “biyuan” and the dialectical classification criteria for “exogenous wind-heat syndrome.” ③ Age 25–65 years. ④ There were no contraindications to surgery and no previous nasal surgery. ⑤ Patients who were informed and voluntarily participated in this research. ⑥ There was no obvious abnormality in the electrocardiogram, blood test, etc.

### 2.3. Exclusion Criteria

① Patients with nasal cavity structural deformity, nasal cavity and sinus tumors, nasal adenoid hypertrophy, severe nasal septum deviation, or fibrous hyperplasia. ② Patients with respiratory infections, immune system diseases, or other serious primary diseases of the heart, brain, liver, kidney, hematopoietic system, etc. ③ Patients with severe mental disorders or mental illness. ④ Patients who had received hormone medication within 1 month before enrollment or drug contraindications. ⑤ Pregnancy, pregnancy intention, and breastfeeding women. ⑥ Combined with other allergic diseases.

### 2.4. Elimination and Fall-Off Criteria

① Patients with poor treatment compliance. ② Patients with severe complications or major adverse reactions during treatment. ③ Patients who were lost during the follow-up period. In this study, 2 cases fell off during the follow-up period in the control group, and 3 cases fell off during the follow-up period in the study group. A total of 107 cases were completed.

### 2.5. Treatment Method

The control group was treated with ESS according to the Messerklinger method. That is, after general anesthesia, the patient's sieve bleb was opened, and then, the patient's nasal polyps were removed with a dynamic system and polyp forceps; then, depending on the patient's condition, the uncinate process and ethmoid vesicles were removed, the maxillary sinus was widened, the different degrees of diseased tissue were exposed and removed properly, and when the operation was over, the absorbable Naxi cotton was full with the wound to stop bleeding. After surgery, levofloxacin capsules (Yangtze River Pharmaceutical Group Co., Ltd., National Medicine Standard H19990051, specification 0.1 g*∗*6 tablets, usage and dosage: 0.2 g/time, 2 times/d) were given orally, budesonide nasal spray (Shanghai Johnson Pharmaceutical Co., Ltd., National Medicine Standard J20180023, specification 64 *μ*g*∗*120 sprays/bottle, usage and dosage: 2 sprays/time, 2 times/d) was given, and normal saline was given to rinse the nasal cavity, etc.

The research group was administered with Xinyi Biyan Pill (Dongguan Asia Pharmaceutical Co,, Ltd., National Medicine Standard Z44021948, specification: 3 g*∗*9 bags, usage and dosage: 3 g/time, 3 times/d) after the operation on the abovementioned basis. The treatment effects were compared after 3 months of continuous treatment in the two groups.

### 2.6. Observe Indicators

① The clinical efficacy of the two groups after treatment was observed. Among them, after treatment, the patient's clinical symptoms disappeared, and endoscopic examination showed that the patient's sinus ostium was well opened, which was effective; after treatment, the patient's clinical symptoms were relieved, and endoscopic examination showed that the patient's sinus cavity area edema, which was getting better; after treatment, the patient's clinical symptoms and nasal endoscopy were not improved, which was invalid [10]. Total effective rate = (effective + get better) number of people/total number of people × 100%.
② The symptom relief time of nasal congestion and runny nose, hyposmia, mucosal edema, and disappearance of vesicles in the two groups after treatment were observed.
③ The fasting venous blood of the two groups was collected, and enzyme-linked immunosorbent assay (ELISA) was used to detect serum inflammatory factors' (C-reactive protein (CRP), interleukin-6 (IL-6), and interleukin-8 (IL-8)) expression level and immune function indicators' (total immunoglobulin E (TIgE), eosinophil cationic protein (ECP), CD3^+^, CD4^+^, and CD4^+^/CD8^+^) expression level before and after treatment.
④ The recurrence rate of the CRS after 1 year of treatment in the two groups was recorded.

### 2.7. Statistical Methods

The SPSS 22.0 software was used, the counting data were expressed as (%), and the comparison was performed by the *χ*^2^ test, and the measurement data were expressed as ($\bar{x}$ ± *s*), and *t* analysis was carried out for comparison. *P* < 0.05 indicated that the difference was statistically significant.

## 3. Results

### 3.1. Comparison of Clinical Efficacy between the Two Groups

After treatment, the total clinical effective rate of the study group (92.98%) was significantly higher than that of the control group (78.00%) (*P* < 0.05), as shown in Table 2.

### 3.2. Comparison of Clinical Symptom Remission Time between the Two Groups

After treatment, the symptom relief time of nasal congestion and runny nose, hyposmia, mucosal edema, and vesicle disappearance in the study group was shorter than that in the control group (*P* < 0.05), as shown in Figure 1.

### 3.3. Comparison of the Expression Levels of Serum Inflammatory Factors between the Two Groups

After treatment, the expression levels of serum CRP, IL-6, and IL-8 in the two groups were significantly lower than those before treatment, and the study group was significantly lower than the control group (*P* < 0.05), as shown in Figure 2.

### 3.4. Comparison of Various Indicators of Serum Immune Function between the Two Groups

After treatment, the expression levels of serum TIgE and ECP of the two groups were significantly lower than those before treatment, and the expression levels of serum CD3^+^, CD4^+^, and CD4^+^/CD8^+^ were significantly higher than those before treatment, and compared with the control group, the changes of the study group were significant (*P* < 0.05), as shown in Figure 3.

### 3.5. Comparison of the Recurrence Rate of CRS between the Two Groups after 1 Year of Treatment

After 1 year of treatment, the recurrence rate of CRS in the study (1.79%) was significantly lower than that of the control group (12.00%) (*P* < 0.05), as shown in Figure 4.

## 4. Discussion

CRS is one of the most difficult diseases in the clinical diagnosis and treatment of otolaryngology. The disease is lingering and difficult to cure. The impact on the quality of life of patients is no less than that of other chronic respiratory diseases such as asthma, chronic bronchitis, and chronic obstructive pulmonary disease. It has brought a heavy economic burden to the patient's family, society, and government. In terms of pathogenesis, the industry generally believes that the occurrence of CRS is the result of multiple factors such as abnormal anatomical structures of the nasal cavity and paranasal sinuses, disorders of the mucociliary transmission system, disorders of the sinus microbial flora, allergies, deficiencies in immune function, accompanying diseases, and genetic polymorphisms. [11, 12]. In terms of clinical classification, it can be divided into two phenotypes, CRS with nasal polyps (CRSwNP) and CRS without nasal polyps (CRSsNP), and four pathological types, neutrophil infiltration, eosinophil infiltration, lymphocyte/plasma cell infiltration, or mixed [13]. In view of the complex pathogenesis of the disease, diverse clinical manifestations, and different prognosis, it has brought great challenges to the diagnosis and treatment of clinicians. Among the existing treatment methods, ESS is the most common surgical intervention method. It can effectively remove the diseased mucosa and preserve the normal mucosa. However, there are still problems such as nasal mucosal adhesion, inflammatory edema, and immune function defects after the operation, and its effect on the improvement of olfactory dysfunction in patients has been controversial. Therefore, it is necessary to supplement with anti-inflammatory, immune enhancement, antiallergic, and nasal orifice drugs after surgery to enhance and consolidate the efficacy and improve the prognosis [14].

According to the guidelines, for the treatment of CRS, symptomatic treatments such as oral macrolides and nasal glucocorticoids can be used to reduce inflammation and allergies and improve nasal symptoms. However, combined with clinical reality, whether it is for CRSwNP or CRSsNP, the effective rate of drug treatment is generally less than 50%, and even if combined with ESS surgical treatment, more than 20% of patients still need to undergo secondary surgery. In recent years, integrated traditional Chinese and Western medicine has shown great advantages in the treatment of this disease. CRS belongs to the category of “biyuan” in Chinese medicine. Its occurrence is closely related to the deficiency of lung qi, the lack of solid body surface, the invasion of wind-heat and evil toxin or wind-cold, the stagnation of heat for a long time, the obstruction of lung meridian, the invasion of evil toxin, and the stagnation of nose orifices, or spleen meridian damp-heat, gallbladder-heat offense, and loss of righteousness. Therefore, the treatment can start with dispelling wind and relieving internal heat or fever, anti-inflammatory, and detoxification. Xinyi Biyan Pill is one of the commonly used drugs in our department for treating cold nasal congestion, allergic rhinitis, chronic rhinitis, and headache, which belongs to wind-heat syndrome in recent years. Its curative effect is accurate, and it is widely used. However, there is still a lack of research reports on the effect of the drug on CRS patients. The medicine ingredients of this medicine contain 13 Chinese herbal medicines such as Xin Yi, *Xanthium*, mint, *Chrysanthemum*, parsnip, *Angelica dahurica*, *Perilla* leaves, coriander, patchouli, *Houttuynia cordata*, Radix Isatidis, trigeminal bitter, and licorice. Among them, Xin Yi and Xanthium are pungent and warm and divergent in nature and have become the monarch medicine. Both are aromatic and transparent, and their characteristics are transmitted upwards, and both have the effects of dispelling wind evil, promoting clearing yang, removing dampness, and clearing nasal orifices. Mint evacuates wind and heat and clears the head and eyes; *Chrysanthemum* evacuates wind and heat, clears heat, and detoxifies; parsnip dispels wind and relieves the surface, dehumidifies, and relieves pain; *Angelica dahurica* dispels pus to relieve orifice, dispels wind, and relieves pain; *Perilla* leaves relieve the surface and promote qi; together, they are used as minister medicine to assist the monarch medicine to enhance the effects of dispelling wind and heat, getting through the orifices, and relieving pain. Accompanied by fragrant coriander, patchouli clears turbid and nose orifices; *Houttuynia cordata*, Radix Isatidis, and trigeminal bitter clear heat and detoxify, reduce swelling and pain, to enhance the efficacy of the monarch medicine and the minister medicine to clear away heat and toxins, reduce dampness and turbidity, and clear the nose orifices. Licorice can not only clear away heat and toxins but also reconcile various medicines, so it is an adjuvant medicine. Combination of all medicines has the effects of dispelling wind, clearing orifice, clearing heat, and detoxification.

In this study, Xinyi Biyan Pill was applied to the adjuvant treatment of CRS patients after ESS. The results showed that, after treatment, the total clinical effective rate (92.98%) of the study group was significantly higher than that of the control group (78.00%) (*P* < 0.05). After treatment, the time to relieve symptoms of nasal congestion and runny nose, hyposmia, mucosal edema, and vesicle disappearance in the study group was shorter than that in the control group (*P* < 0.05). It shows that Xinyi Biyan Pill has a significant clinical effect in adjuvant treatment of CRS and can effectively relieve the symptoms and signs of CRS patients. According to the report of Bochner and Stevens [15], the inflammatory changes of nasal mucosa caused by inflammatory cells and related mediators are the important pathophysiological basis for the occurrence of different phenotypes and subtypes of CRS. Among them, CRP is an important acute phase response protein that is positively correlated with the degree of inflammation in the body. IL-6 is a pleiotropic inflammatory cytokine produced by monocytes, vascular endothelial cells, etc., when inflammation or infection occurs in the body; it participates in immune response regulation and cell damage together with other cytokines [16]. IL-8 is a chemokine that is secreted by Th1 cells, and it has the effect of chemotaxis and activation of inflammatory cells such as neutrophils and mediates immune pathological damage and local inflammation [17]. After treatment in this study, the expression levels of serum CRP, IL-6, and IL-8 in the two groups were significantly lower than those before treatment, and the study group was significantly lower than the control group (*P* < 0.05). It indicates that the anti-inflammatory mechanism of Xinyi Biyan Pill in the treatment of CRS may be related to the inhibition of the expression of serum CRP, IL-6, and IL-8. In addition, allergies are also of great significance in the continuous process of CRS [18]. Serum TIgE and ECP are both important detection indicators that reflect the degree of allergies in the body. Among them, TIgE's synthesis can be significantly increased under the stimulation of certain allergens. ECP is a specific indicator that can reflect the degree of eosinophil activation. Both are highly expressed in the serum content of CRS patients [19, 20]. After treatment in this study, the serum TIgE and ECP expression levels of the two groups of patients were significantly lower than before treatment, and the study group was significantly lower than the control group (*P* < 0.05). It shows that Xinyi Biyan Pill can reduce the degree of allergy in CRS patients, thereby inhibiting disease progression. In addition, the body of CRS patients will also show varying degrees of immunosuppression, which may be related to the disorder of secretion and the destruction of the balance mechanism of T-lymphocyte subsets in the disease state [21]. CD3^+^ is an important indicator for maintaining the immune function of the body, CD4^+^ is an important factor for regulating the immune response, and the balance of CD4^+^/CD8^+^ is the key mechanism that mediates immune balance [22]. After treatment in this study, the serum CD3^+^, CD4^+^, and CD4^+^/CD8^+^ expression levels of the two groups of patients were significantly higher than before treatment, and the study group was significantly higher than the control group (*P* < 0.05). It shows that the adjuvant treatment of Xinyi Biyan Pill has a good benign regulatory effect on the T-cell immune response of CRS patients and helps maintain the immune balance mechanism. The results of this study also showed that after 1 year of treatment, the recurrence rate of CRS in the study group (1.79%) was significantly lower than that in the control group (12.00%) (*P* < 0.05). This further suggests that the adjuvant treatment of Xinyi Biyan Pill is an effective way to consolidate the postoperative curative effect of ESS and reduce clinical recurrence in CRS patients.

In summary, Xinyi Biyan Pill has significant clinical effects in adjuvant treatment of CRS patients, which can effectively reduce the expression level of serum inflammatory factors, improve the body's immune function, and prevent short-term recurrence. It is worthy of clinical promotion.

## Figures and Tables

**Figure 1:** Comparison of clinical symptom relief time between the two groups ($\bar{x}$ ± *s* (d)). Note: after treatment in the control group, the symptom relief time of nasal congestion and runny nose, hyposmia, mucosal edema, and vesicle disappearance was (14.23 ± 2.42) d, (24.98 ± 3.64) d, (16.30 ± 3.25) d, and (44.97 ± 6.04) d, respectively. After treatment in the study group, the symptom relief time of nasal congestion and runny nose, hyposmia, mucosal edema, and vesicle disappearance was (8.87 ± 1.73) d, (13.27 ± 2.21) d, (9.41 ± 1.56) d, and (23.23 ± 4.79) d, respectively. ^*∗*^The comparison with the control group, *P* < 0.05.

**Figure 2:** Comparison of the expression levels of serum inflammatory factors between the two groups ($\bar{x}$ ± *s* (pg/L)). (a) Serum CRP expression levels. Its expression levels before and after treatment in the control group were (10.43 ± 3.26) pg/L and (5.20 ± 1.13) pg/L, and its expression levels before and after treatment in the study group were (10.07 ± 3.12) pg/L and (2.87 ± 0.68) pg/L, respectively. (b) Serum IL-6 expression levels. Its expression levels before and after treatment in the control group were (14.61 ± 3.94) pg/L and (8.83 ± 1.02) pg/L, and its expression levels before and after treatment in the study group were (14.75 ± 4.07) pg/L and (4.66 ± 0.95) pg/L, respectively. (c) Serum IL-8 expression levels. Its expression levels before and after treatment in the control group were (137.29 ± 18.04) pg/L and (82.68 ± 6.73) pg/L, and its expression levels before and after treatment in the study group were (138.15 ± 18.23) pg/L and (64.40 ± 5.71) pg/L, respectively. ^*∗*^The comparison with the same group before treatment, *P* < 0.05; ^#^the comparison with the control group after treatment, *P* < 0.05.

**Figure 3:** Comparison of various indicators of serum immune function between the two groups ($\bar{x}$ ± *s*). (a) Serum TIgE expression levels. Its expression levels before and after treatment in the control group were (84.62 ± 8.35) kU/L and (64.37 ± 7.25) kU/L, and its expression levels before and after treatment in the study group were (85.13 ± 8.41) kU/L and (58.53 ± 7.39) kU/L, respectively. (b) Serum ECP expression levels. Its expression levels before and after treatment in the control group were (7.17 ± 1.50) ng/L and (4.98 ± 1.06) ng/L, and its expression levels before and after treatment in the study group were (7.20 ± 1.52) ng/L and (4.26 ± 0.81) ng/L, respectively. (c) Serum CD3^+^ expression levels. Its expression levels before and after treatment in the control group were (51.86 ± 5.33) % and (57.69 ± 5.24) %, and its expression levels before and after treatment in the study group were (52.17 ± 5.32) % and (66.26 ± 5.41) %, respectively. (d) Serum CD4^+^ expression levels. Its expression levels before and after treatment in the control group were (30.89 ± 5.50) % and (33.91 ± 4.67) %, and its expression levels before and after treatment in the study group were (30.89 ± 5.50) % and (33.91 ± 4.67) %, respectively. (e) Ratio of CD4^+^/CD8^+^. Its expression levels before and after treatment in the control group were (1.08 ± 0.22) and (1.17 ± 0.21), and its expression levels before and after treatment in the study group were (1.10 ± 0.21) and (1.44 ± 0.24), respectively. ^*∗*^The comparison with the same group before treatment, *P* < 0.05; ^#^the comparison with the control group after treatment, *P* < 0.05.

**Figure 4:** Comparison of the recurrence rate of CRS between the two groups after 1 year of treatment (*n* (%)). Note: there were 6 cases of CRS recurrence after 1 year of treatment in the control group and 1 case of CRS recurrence in the study group after 1 year of treatment. ^*∗*^There was a statistically significant difference in the recurrence rate of CRS between the control group and the study group after treatment (*χ*^2^ = 4.573, *P*=0.032).

**Table 1:** Comparison of two groups of general information (*n* (%), $\bar{x}$ ± *s*).

Types	Control group (*n* = 52)	Study group (*n* = 60)	*χ*^2^/*t*	*P*
Gender			0.061	0.804
Male	30 (57.69%)	36 (60.00%)		
Female	22 (42.31%)	24 (40.00%)		
Age (year old)	36.52 ± 8.69	35.94 ± 9.07	0.344	0.731
Course of disease (years)	5.22 ± 2.13	5.19 ± 2.15	0.074	0.941
Nasal polyp			0.106	0.745
Yes	27 (51.92%)	33 (55.00%)		
No	25 (48.08%)	27 (45.00%)		

**Table 2:** Comparison of clinical efficacy between the two groups (*n* (%)).

Group	*n*	Effective	Get better	Invalid	Total effective rate
Control group	50	32 (64.00)	7 (14.00)	11 (22.00)	39 (78.00)
Study group	57	48 (84.21)	5 (8.77)	4 (7.02)	53 (92.98)
*χ* ^2^					4.960
*P*					0.026

## Data Availability

The data used and/or analyzed in the current research can be obtained from the corresponding author according to reasonable requirements.
